# Effects of the epigenetic drug MS-275 on the release and function of exosome-related immune molecules in hepatocellular carcinoma cells

**DOI:** 10.1186/2047-783X-18-61

**Published:** 2013-12-23

**Authors:** Wenhua Xiao, Weiwei Dong, Caihong Zhang, Gaowa Saren, Paili Geng, Huixia Zhao, Quiwen Li, Jianhua Zhu, Guanghui Li, Shufang Zhang, Ming Ye

**Affiliations:** 1 The First Affiliated Hospital, PLA General Hospital, Fucheng Road 51, Beijing, China; 2 Department of Immunology, Medical College of Qinghai University, No.16 Kunlun Road, Xining 810001, Qinghai Province, China; 3 Department of Histology and Embryology, Inner Mongolia Medial College, Inner Mogolia Autonomous Region, Hohhot 010010, China

**Keywords:** Exosomes, HepG2, HSP70, MICA, MICB, NK cell

## Abstract

**Background:**

Tumor-derived exosomes have been viewed as a source of tumor antigens that can be used to induce anti-tumor immune responses. In the current study, we aim to investigate the regulatory effect of the epigenetic drug MS-275 on hepatoma G2 (HepG2) cell-derived exosomes, especially for their immunostimulatory properties and alteration of some non-specific immune protein expression, such as heat shock protein (HSP) 70, major histocompatibility complex (MHC) class I polypeptide-related sequence A (MICA) and MICB.

**Methods:**

MS-275 was used to modulate the secretion of exosomes in human HepG2 cells, and exosomes from untreated HepG2 cells served as negative controls. RT-PCR was used to test the expression of HSP70, MICA and MICB in HepG2 cells. Immunogold labeling of exosomes and western blotting analysis were carried out to compare the expression of HSP70, MICA and MICB proteins in exosomes with or without MS-275 treatment. A natural killer (NK) cell cytotoxicity assay and peripheral blood mononuclear cell (PBMC) proliferation assay were used to evaluate the effect of MS-275 on the immunostimulatory ability of exosomes.

**Results:**

Immunogold labeling and western blot analysis showed that modification of MS-275 increased the expression of HSP70 and MICB in exosomes. RT-PCR showed the mRNA levels of HSP70 and MICB were upregulated in HepG2 cells and were consistent with their protein levels in exosomes. The exosomes modified by MS-275 could significantly increase the cytotoxicity of NK cells and proliferation of PBMC (*P* < 0.05).

**Conclusions:**

The non-specific immune response of exosomes derived from HepG2 cells could be enhanced with treatment by the histone deacetylase inhibitor (HDACi) drug MS-275; this could provide a potential tumor vaccine strategy against liver cancer.

## Background

Exosomes are small membrane-bound particles with a diameter of 30 to 100 nm; exosomes can be released from both normal and diseased cells, such as neoplastic cells, to the blood and other bodily fluids [1-3]. They contain signal proteins and/or peptides, microRNAs, mRNAs, and lipids [4,5], and, after release from diseased or normal cells, some exosomes are transported to distant sites by blood [6,7]. Studies have shown that exosomes secreted by tumor cells have immunosuppressive and pro-cancer activities [3,8]; both *in vivo* and *in vitro* evidence has showed that exosomes derived from tumor cells can augment an anti-tumor response [9,10]. However, the capacity of tumor-derived exosomes in the cellular immune response against tumors is limited by numerous factors, including the heterogeneity of tumor antigens, the type and molecular chaperone of immune molecules in different tumor cells, the insufficient expression of tumor-associated antigens and immune molecules, the inhibited immune cell proliferation by tumor-derived exosomes, and downregulated NKG2D ligand expression at the tumor cell surface which influences the activity of natural killer (NK) cells and their cytotoxicity to tumor cells [11-13].

MS-275 is one of the histone deacetylase inhibitor (HDACi) drugs which is commonly used as an epigenetic drug to upregulate tumor specific antigens such as human leukocyte antigen-I, human leukocyte antigen-II, co-stimulatory molecule B7, and immune adhesion molecules. MS-275 could enhance the specific and non-specific anti-tumor immune reaction. In this study, we attempted to explore the effects of MS-275 on the release and function of exosome-related immune molecules in hepatoma G2 (HepG2) cells.

## Methods

### Preparation of peripheral blood mononuclear cells and natural killer cells

Following approval from our hospital ethics committee, 20 ml peripheral blood samples were collected into a 50-ml CPT cell preparation tube (Becton Dickinson, Cowley, UK) from healthy donors who signed consent forms. Peripheral blood mononuclear cells (PBMCs) were isolated by Ficoll gradient centrifugation as previously described [14]. After washing in PBS, cells were resuspended in RPMI 1640 medium at a concentration of 1 × 10^7^/ml.

Peripheral blood NK cells were negatively selected from PBMCs by magnetic sorting using the Mini MACS NK isolation kit (Miltenyi Biotech, Shanghai, China). Isolated NK cells were activated by phytohemagglutinin (PHA;10 ng/ml; Sigma-Aldrich, St Louis, MO, USA) and IL-2 (1,000 IU/ml) in RPMI 1640 medium supplemented with 10% FCS.

### Isolation of exosomes from culture supernatants with or without MS-275

The human HepG2 cell line (JCRB1054) was obtained from Beijing Cancer Research and Prevention Institute, Beijing, China. Cells were cultured in DMEM supplemented with 10% FBS, 100 U/ml penicillin, and 100 μg/ml streptomycin at 37°C in an atmosphere of 5% CO_2_. MS-275 was purchased from Sigma-Aldrich.

Log phased HepG2 cells were plated into dishes at a density of 3 × 10^4^/ml. After 24-hour culture, MS-275 (1 × 10^-6^ mol/l) was added. PBMCs treated with PHA served as the blank control. After incubation for 72 hours, culture media was collected and sequentially centrifuged at 300 × g at 4°C for 3 minutes, floating cells were removed, and then centrifuged at 2,000 × g for 15 minutes at 4°C and at 12,000 × g at 4°C for 35 minutes. Cell debris was then removed. Supernatants were collected and passed through a 0.22 μm filter. Exosomes were isolated by ultra-centrifugation at 120,000 × g at 4°C for 2 hours, and quantified by measuring their protein concentration with a BCA assay (μg/ml). Exosomes pellets were stored at −80°C until use.

### Electron microscopic characterization and immunogold labeling of exosomes

A total of 20 to 30 μl prepared exosomes were loaded onto a copper net. Following air drying, 30 μl phosphotungstic acid solution (pH 6.8, 20 ml/l) was added and a negative staining was performed at room temperature for 1 minute. After drying at room temperature about 10 minutes, staining signals of the microcapsule membrane structure (30 to 80 nm) were observed under a photographic transmission electron microscope.

For immunogold labeling, exosomes were applied to formvar carbon-coated copper grids and incubated with rabbit anti-human heat shock protein (HSP)70 monoclonal antibody (1:50 diluted, StressGen Biotechnologies Corporation, British Columbia, Canada), rabbit anti-human anti-major histocompatibility complex (MHC) class I polypeptide-related sequence A (MICA) antibody and rabbit anti-human anti-MICB monoclonal antibody (1:100 diluted, Biolegend, Sandiego, CA, USA), respectively, at room temperature for 1 hour. Incubation with PBS served as a blank control. Following washing in PBS, exosomes were incubated with 20 μl protein A immunogold (SPA) (1:15 diluted) at room temperature for 30 minutes. A negative dye containing 15 μl uranyl acetate was performed at room temperature for 30 seconds. Positively labeled exosomes were seen as vesicles containing black colloidal gold particles under the transmission electron microscope. The numbers of exosomes were counted in 10 random fields (1000 nm × 700 nm). Counting was repeated five times and the average was calculated for each of the specimens.

### ^3^H-TdR incorporation assay of peripheral blood mononuclear cell proliferation

PBMCs were plated into a 96-well plate at a concentration of 5,000 cells/well in RPMI 1640 medium supplemented with 10% FBS; streptomycin and penicillin were added at a final concentration of 50 μg/l with or without PHA (100 μl loaded). In total, three groups were involved. The wells without exosomes served as controls, and the other two groups had either normal exosomes added or exosomes modified with MS-275, respectively (final exosome concentration 10 μg/ml). After culture at 37°C in an atmosphere of 5% CO_2_ overnight, H^3^-TdR was added to each well at a concentration of 3.7 × 10^4^ Bq. Following an incubation for 6 hours, 1 mol/l NaOH was used to break the cell membrane. Scintillation fluid and the quenching agent were added, and the H^3^-TdR incorporation was quantified as counts per minute (CPM) on a beta liquid scintillation counter (PerkinElmer Life Sciences, Waltham, MA, USA).

### RNA isolation and RT-PCR

After incubation with MS-275 for 3 days, HepG2 cells were washed and prepared for analysis. Total RNA was isolated using the RNeasy Micro Kit (Qiagen, Hilden, Germany). Single-strand cDNA was synthesized and HSP70, MICA and MICB were amplified using the following specific primers (Eurofins MWG Operon, Ebersberg, Germany): HSP70 forward 5′-TGTGGCTTCCTTCGTTATTGG-3′ and reverse 5′-GCCAGCATCATTCACCACCAT-3′; MICA sense, 5′-CAGGGACTTGACAGGGAAC-3′ and antisense, 5′-CCTCTCCTCGGCAAATCCT-3′; MICB sense, 5′-ACCGAGGACTTGACAGAGA-3′ and antisense, 5′-CCGCTGATGTTTTC CTTCT-3′; and reverse: 5′-CACCTTGCCGTGTTGGAA-3′ GAPDH forward: 5′-CCACTCCTCCACCTTTGAC-3′ and reverse: 5′-ACCCTGTTGCTGTAGCCA-3′. The PCR products were separated on 2% agarose gel and visualized with ethidium bromide. GADPH served as a control.

### Western blotting analysis

Protein electrophoresis was performed as previously described [15]. After transfer, membrane blots were stained with Ponceau S to verify quality of transfer and equal loading. Blots were probed for HSP70 and MICA and MICB using primary anti-HSP70 (1:500, StressGen) and MICA and MICB (Santa Cruz Biotechnology, Santa Cruz, CA) antibodies, respectively; horseradish peroxidase-conjugated anti-goat served as a secondary antibody (Amersham/GE, Piscataway, NJ, USA). Specific immunoreactive signals were developed with a chemiluminescent agent (Pierce, Rockford, IL, USA). Densitometric analysis was performed as previously described [16].

### Cytotoxicity assay

An AlamarBlue based one-step fluorimetric assay was performed as previously described [17]. Briefly, prepared normal exsomes and MS-275 modified exosomes (10 μg/ml) were added to the target HepG2 cells in 96-well flat-bottomed plates, and effector cells (NK cells) were added; mixed effector and target cells were at ratios of 1:5, 1:10, 1:20, and 1:40, respectively. The mixtures were incubated with AlamarBlue in a humidified environment with 5% CO_2_ at 37°C overnight. The fluorescent signals of the AlamarBlue were read by a Synergy HT plate reader (Biotek, Winooski, VT, USA) at excitation of 530 nm and emission of 590 nm, respectively. The cytotoxicity of NK cell was calculated using the following formula:

$$\begin{array}{c} \mathrm{NK}\;\text{cell}\;\text{cytotoxicity}\;\left(\%\right)=\left(\mathrm{AF}\;\mathrm{of}\;\text{observation}\;\text{group}–\mathrm{AF}\;\mathrm{of}\;\text{target}\;\text{cells}–\mathrm{AF}\;\mathrm{of}\;\text{effector}\;\text{cells}\right)/\\ \;\left(\mathrm{AF}\;\mathrm{of}\;\text{fully}\;\mathrm{lysis}\;\text{target}\;\text{cells}–\mathrm{AF}\;\mathrm{of}\;\text{target}\;\text{cells}\right)\times 100\% \end{array}$$

where AF is the average fluorescence units.

### Statistical analysis

Data were analyzed by chi-square test using SPSS 19.0 software IBM, Chicago, IL, USA. Differences were considered significant at *P* < 0.05.

## Results and discussion

### Electron microscopic characteristics of exosomes

The exosomes secreted from HepG2 cells were round or oval membrane microcapsules with a diameter of 30 to 80 nm when observed under an electron microscope; the composition within the membrane showed a low electronic density (Figure 1A). We counted the average exosome number treated with or without MS-275, and the exosomes secreted by HepG2 cells increased greatly (*P* < 0.05) after treatment with MS-275 (Figure 1B). The immunogold labeling showed black granular colloidal gold signals existed in the capsular membrane and cavity. Compared with untreated HepG2 cells, MS-275-treated HepG2 cells expressed significantly higher (*P* < 0.001) levels of HSP70 and MICB-positive colloidal gold particles in exosomes (Figure 2); although we observed relative high levels of MICA after treatment with MS-275, there was no difference when compared with untreated exosomes. In untreated cells, the number of HSP70-positive colloidal gold particles was much higher than MICA- and MICB-positive particles.

**Figure 1:** **The electron microscope observation result of exosomes secreted from hepatoma G2 cells. (A)** The microcapsule of exosomes have a diameter of 30 to 80 nm. **(B)** Column comparison of exosome expression with or without MS-275.

**Figure 2:** **The comparison of immunogold labeling of hepatoma G2 cells treated with or without MS-275.** After treatment with MS-275, heat shock protein (HSP)70, MICA, and MICB molecular colloidal gold particles increased in exosomes with statistical significance (*P* < 0.01). **(A)** HSP70 protein without drug. **(B)** HSP70 protein treated with drug. **(C)** MICA protein without drug. **(D)** MICA protein treated with drug. **(E)** MICB protein without drug. **(F)** MICB protein treated with drug.

### Effect of MS-275 on peripheral blood mononuclear cell proliferation

The CPM value decreased in the exosomes modified by drug group (19,411 ± 786.63) when compared with the value in the blank control group (23,974 ± 2,024.31), but the difference between these two groups failed to reach a significant level (*P* > 0.05). In contrast, the CPM value was decreased significantly in the group of exosomes without drug modification (3,863 ± 20.88) when compared with the value in the blank control group (*P* < 0.001) and the exosomes modified by drug group (*P* < 0.05).

### MS-275 induced elevated expression of heat shock protein 70, MICA, and MICB in hepatoma G2 cells

After treatment with MS-275, the mRNA expression of HSP70, MICA, and MICB were all upregulated in HepG2 cells, compared to cells without treatment by MS-275. The relative expression of HSP70, MICA, and MICB was upregulated by 3.4-, 3.6- and 2.8-fold, respectively (Figure 3).

**Figure 3:** The mRNA expression of heat shock protein (HSP)70, MICA and MICB in hepatoma G2 cells.

### Western blotting analysis results

Consistent with mRNA expression, western blotting analysis showed the specific protein bands of HSP70 (147 kDa), MICA (73 kDa) and MICB (47 kDa) in the HepG2 cell-derived exosomes (Figure 4). MS-275 modification significantly increased MICB and HSP70 protein in the exosomes of HepG2 cells compared to those without MS-275 treatment (*P* < 0.05).

**Figure 4:** **Comparison expression of heat shock protein (HSP)70, MICA and MICB protein with or without MS-275. (A)** Western blot showing the protein band of HSP70, MICA and MICB at the molecular weights of 147, 73 and 47 kDa, respectively. EMD, exosomes with drug modification; EWD, exosomes without drug modification. **(B)** Histogram comparison; after treatment with MS-275, the expression of MICA, MICB and HSP70 in HepG2 cell exosomes (EMD) increased significantly compared with untreated cells (EWD).

### Natural killer cell cytotoxicity

We evaluated the cytotoxicity of NK cells against HepG2 cells at various NK/HepG2 cell ratios with normal or MS-275 modified exosomes. The results are presented in Table 1. As the NK/HepG2 cell ratio increased, the dead HepG2 cells increased. MS-275 significantly increased the cytotoxicity of NK cells at the same effector/target cell ratio (*P* < 0.05).

**Table 1:** Percentage of hepatoma G2 cells killed by natural killer cells at various effector: target cell ratios with or without MS-275 modification

	**Effector cell (NK cells): target cell ratios**			
	**5:1**	**10:1**	**20:1**	**40:1**
EWD group (%)	1. 69 ± 0.13	2. 47 ± 0. 84	5. 21 ±1. 07	5. 77 ± 0. 83
EMD group (%)	25. 32 ± 1. 31^*^	42. 27 ± 1.67^*^	57. 53 ± 2.13^*^	70.21 ± 3. 01^*^

*P < 0.05 compared with EWD group. EMD: exosomes with drug modification; EWD, exosomes without drug modification; NK, natural killer.

Exosomes are vesicles formed by ‘inward/reverse budding’ of the limiting membrane of the multivesicular bodies in the late endocytic compartment that are released upon the fusion of multivesicular bodies with the plasma membrane [18,19]. Exosome proteins derived from the tumor cell membrane are rich in tumor antigen chaperone molecules such as HSP70, 80, 90 and MHC class I molecules. HSP70 originated from tumor exosomes can selectively activate NK cell activity, thus leading to the migration and proliferation of tumor cell and augmentation of an immune response [20]. Due to their molecular chaperone properties, HSPs can bind tumor-specific peptides and deliver them deep into the antigen-processing pathways of antigen-presenting cells. In this way, HSP-based vaccines can activate tumor-specific immunity, trigger the proliferation and cytotoxic T lymphocyte capabilities of cancer-specific CD8^+^ T cells, and inhibit tumor growth [21]. However, the immune stimulatory activity of exosomes in tumor cells is dependent on their expression level. Moreover, tumor-derived exosomes lack antigen presentation stimulators such as T-cell-activating protein, latent membrane protein and Tapasin; as a result, their tumor immunosuppressive activity is substantially compromised [22].

The extent of exosome secretion in different cell types can be modulated by either ligand cognition or stresses. For example, radiation treatment is able to increase the level of exosomes secreted by tumor cells, a process possibly involving the activation of p53 and the subsequent upregulation of the trans-membrane protein tumor suppressor-activated pathway 6 [23,24]. HDACi exert their effects predominantly by altering histone acetylation, which is normally controlled by a balance between histone deacetylases and histone acetyltransferases [25]. Increased histone acetylation induced by HDACi results in activation of the genes responsible for: 1) generating an intracellular pro-apoptotic milieu [26], 2) increasing surface expression of TNF, super-family death receptors like Fas, TNF-related apoptosis-inducing receptor and TNF-receptors [27], 3) increasing the expression of MHC molecules and other molecules involved in antigen processing and presentation [22,28], and 4) increasing expression of tumor antigens recognized by cytotoxic T lymphocytes and ligands for NK activating receptors [29].

In our study, we found MS-275 was able to increase the secretion of MICB and HSP70 in exosomes secreted by HepG2 cells significantly. We also observed that MS-275 modification could attenuate the inhibitory effect of naive exosomes on the cytotoxicity of NK cells, possibly through upregulating the expression of the MICA, MICB, and HSP70 on the tumor cell surface. These observations were consistent with the results of electron microscopic assessment.

## Conclusion

In conclusion, soluble immunoregulatory molecules in the exosomes secreted by HepG2 cells have a significant inhibitory effect on lymphocyte proliferation. MS-275 modified exosomes enhance the cytotoxic effect of NK cells significantly through upregulating the expression of MICA, MICB and HSP70. Our observations suggest that HDACi-modified tumor cell-derived exosomes may function as potential tumor vaccines against liver cancer. We only observed one HDACi drug (MS-275) and one tumor cell line (HepG2); therefore, it is difficult to conclude that this conclusion is universally represented. An in-depth study is therefore needed, but our study can provide some reference for similar research.

## Abbreviations

CPM: Counts per minute; DMEM: Dulbecco’s modified Eagle’s medium; FBS: Fetal bovine serum; FCS: Fetal calf serum; HDACi: histone deacetylase inhibitor; HepG2: Hepatoma G2; HSP: heat shock protein; IL: Interleukin; MHC: Major histocompatibility complex; MICA: MHC class I polypeptide-related sequence A; MICB: MHC class I polypeptide-related sequence B; NK: natural killer; PBMC: Peripheral blood mononuclear cell; PBS: Phosphate-buffered saline; PHA: Phytohemagglutinin; RT-PCR: Reverse transcriptase polymerase chain reaction; TNF: Tumor necrosis factor.

## Competing interests

The authors declare that they have no competing interests.

## Authors’ contributions

WX and CZ defined the research theme. GS and PG designed methods and experiments, carried out the laboratory experiments, analyzed the data, and interpreted the results. HZ and WD co-designed the dispersal and colonization experiments. QL and JZ co-worked on associated data collection and their interpretation. GL, SZ and MY co-designed experiments, discussed analyses, interpretation, and presentation. All authors read and approved the final manuscript.
